# Estimation of Nuclear Medicine Exposure Measures Based on Intelligent Computer Processing

**DOI:** 10.1155/2021/4102183

**Published:** 2021-09-27

**Authors:** Junfeng Wang, Fangxiao Wang, Yue Liu, Yuanfan Xu, Jiangtao Liang, Ziming Su

**Affiliations:** ^1^Hangzhou Universal Medical Imaging Diagnostic Center, Hangzhou,, Zhejiang 31000, China; ^2^Hangzhou Dianzi University, Hangzhou,, Zhejiang 31000, China

## Abstract

This paper provides an in-depth discussion and analysis of the estimation of nuclear medicine exposure measurements using computerized intelligent processing. The focus is on the study of energy extraction algorithms to obtain a high energy resolution with the lowest possible ADC sampling rate and thus reduce the amount of data. This paper focuses on the direct pulse peak extraction algorithm, polynomial curve fitting algorithm, double exponential function curve fitting algorithm, and pulse area calculation algorithm. The detector output waveforms are obtained with an oscilloscope, and the analysis module is designed in MATLAB. Based on these algorithms, the data obtained from six different lower sampling rates are analyzed and compared with the results of the high sampling rate direct pulse peak extraction algorithm and the pulse area calculation algorithm, respectively. The correctness of the compartment model was checked, and the results were found to be realistic and reliable, which can be used for the analysis of internal exposure data in radiation occupational health management, estimation of internal exposure dose for nuclear emergency groups, and estimation of accidental internal exposure dose. The results of the compartment model of the respiratory tract and the compartment model of the digestive tract can be used to calculate the distribution and retention patterns of radionuclides and their compounds in the body, which can be used to assess the damage of radionuclide internal contamination and guide the implementation of medical treatment.

## 1. Introduction

With the continuous development of nuclear technology, the exposure to ionizing radiation is gradually increasing, and the number of ionizing radiation practitioners is also increasing day by day. Ionizing radiation, also known as nuclear radiation, mainly includes X-rays, *α*-rays, *β*-rays, *γ*-rays, and neutrons. Rays are a high-speed movement of microparticle streams, the process of objects emitting such particle streams is radiation, which can make other atoms, and molecule ionized rays are called ionizing radiation, said to emit ionizing radiation objects for radioactive sources, with radioactive. The main sources of people's exposure to nuclear radiation can be divided into natural radiation and artificial radiation. The Earth is exposed to various types of naturally occurring ionizing radiation every moment; i.e., natural ionizing radiation, generally also known as natural background exposure, is by far the most important source of human exposure to ionizing radiation, with a relatively constant dose rate of irradiation [1]. In recent decades, human exposure to a variety of artificial radiation has been on the rise due to the increase in medical exposures, nuclear power, industrial applications, and the artificial manufacture and use of radionuclides such as nuclear weapons. Among them, the main ones are beta rays, X-rays, and gamma rays [2]. The most widely used in clinical nuclear medicine are single-photon emission computed tomography (SPECT) and positron emission tomography (PET) imaging, which mainly detects gamma rays emitted by radionuclides introduced into the human body and obtains in vivo images, with functional imaging as the main feature, mainly used for metabolic imaging, tumor diagnosis, etc. As our concept of elementary particles continues to change, our understanding of the fundamental forces of nature and the interactions between elementary particles is also evolving [3]. In the process of the gradual deepening of human understanding of the material world, experimental methods and tools have also been gradually improved [4].

While the emergence of clinical nuclear medicine brings great benefits to human health diagnosis and disease treatment, the use of radioisotopes will produce gaseous, liquid, or solid radioactive waste; on the other hand, it is difficult to discharge all radioactive drugs in the body of the patient receiving treatment in a short period. A data processing method that approximates or compares the functional relationship between the coordinates represented by discrete points with a continuous curve. Although the curve obtained by “fitting” cannot guarantee to pass all sample points, it can approximate the true value very well. Therefore, in the practice of clinical nuclear medicine treatment, not only the patients themselves but also the relevant staff and the public may be exposed to additional radiation, potentially posing a certain risk of radiation hazard [5]. For this reason, it is necessary to evaluate the exposure dose and risk assessment of patients and related workers. According to the report, the collective effective dose due to nuclear medicine has tripled in the last decade as the frequency of nuclear medicine diagnostic applications has increased. Reports indicate that nuclear medicine has become the second-largest source of medical exposure after CT scans. In recent years, the world has been developing a study on the trend of dose due to nuclear medicine, but in China, although the frequency of nuclear medicine equipment and treatment has increased significantly in recent years, no study on the collective dose due to nuclear medicine and its trend has been seen, which is not in line with the development of a large country in terms of population and nuclear medicine, so it is necessary to develop a study on the trend of collective dose due to nuclear medicine [6].

During nuclear medicine treatment, radiation exposure to organs or tissues in the patient's body is caused by the presence of radionuclides in the patient's body; therefore, the assessment of internal radiation dose to the patient can be used not only to evaluate the risk of radiation hazards but also to assess the therapeutic effect of certain specific organs or tissues. Internal radiation dosimetry involves not only physics but also radiopharmaceuticals, human-specific biological behavior, and human geometry, which makes the calculation complex and the accuracy of the results poor. Because it is difficult to make in vivo measurements on humans, its dose studies are more of estimation than measurement. There are mainly three different methods for dose estimation, which are the volume element S-value method, the dose point kernel method, and the Monte Carlo calculation method. The dose point kernel method first determines the dose point kernel and then convolutes the source to find the absorbed dose in the corresponding medium. The dose point kernel represents the distribution of the absorbed dose of an isotropic point source in an infinite homogeneous medium, which is essentially a matrix of the absorbed dose rate of a point source of a specific nuclide in a specific medium with the distance from the source, and its physical meaning is the absorbed dose rate at a distance *r* from the point source of unit activity. The formula for calculating the dose point nucleus is generally based on the experimental data fitting correction but also based on Monte Carlo simulation experimental data after correction. Depending on the particle source, it is divided into electron dose point kernel and photon dose point kernel. Comparing the double exponential function fitting of the original waveform and the original waveform fitting without the baseline part, the baseline information cannot be included in the fitting process if the fitting starts from the starting point of the pulse waveform. The dose point kernel method is suitable for the dose calculation of point sources with a nonuniform distribution of activity inhomogeneous media, and the energy range of particles is also required, so its application conditions limit its wide application. Combining the calculation of common external radiation dose rate calculation models and field experimental measurements, we establish the calculation model of external radiation levels for nuclear medicine treatment patients, combine the calculation model established in this study with the possible exposure scenarios of relevant surrounding personnel, project the exposure doses of relevant personnel, and propose specific methods or measures to strengthen the management of radiation protection in conjunction with the relevant regulations of radiation protection.

## 2. Related Work

Pyroelectric dosimeter under the action of radiation will produce charge accumulated in it; the number of accumulated charges can characterize the number of electron-hole pairs produced by radiation, that is, the absorbed dose [7]. Using general pyroelectric dosimeter after wearing a period, using a special readout instrument, by heating or irradiation with bright light, and recording the number of photons released, ideally, the number of photons released, and the number of charges accumulated in it, so the total absorbed dose received during this wearing time can be readout [8]. After reading out the dose, all the accumulated charges can be erased and reused [9]. Pyroelectric dosimeters are passive dosimeters (no power supply required) and are currently the most widely used materials based on LiF, which have a very low rate of decay of accumulated charges escaping over time, have an effective atomic number like that of human soft tissue, and have a lower overresponse to low-energy *X-* and *γ*-rays than materials with higher atomic numbers [10]. Chemiluminescent dosimeter has the advantages of small size, ease of use, and good tissue equivalence, but it can only record the dose received by personnel, the feedback period of up to several months, cannot indicate the dose accumulation in real time, and cannot promptly remind personnel of the dose being too high to change the work style to reduce the dose received by personnel [11]. Currently, a breakthrough has been made in nuclear radiation monitoring systems built on rapidly developing communication technologies [12]. There is a need to layout a lot of equipment and equipment maintenance personnel; the cost is still too high and is very vulnerable to the weather and geographical environment [13]. Therefore, we still cannot meet the needs of users of the nuclear radiation detection system [14]. Along with the development of wireless communication technology, in the acquisition of nuclear radiation data, environmental radiation detector, and gamma energy spectrometer in the introduction of wireless communication technology, compared to the use of wired communication system, to a certain extent to reduce the cost, but we still cannot overcome the many shortcomings of the nuclear radiation detection system [15].

At present, the commonly used equipment for nuclear medicine imaging diagnosis is *γ* camera, SPECT, and PET. SPECT is made by adding a tomographic reconstruction function based on the *γ* camera, so the quality control method of SPECT also includes the quality control method of the *γ* camera. The number of medical institutions carrying out interventional radiology treatment projects and the number of radiologists engaged in interventional radiology work is increasing year by year [16]. With the continuous expansion of the clinical application of interventional radiology and the complexity of the surgery, the characteristics of bedside close operation, long operation time, high irradiation dose, and protection difficulties of interventional radiologists are becoming increasingly prominent. The radiation protection of interventional radiology staff, especially the operators, has attracted widespread attention. Although interventional radiology has brought tremendous benefits to humankind, scientists have also begun to pay attention to the radiation protection issues that arise from it. Among medical diagnostic X-rays, patients and professionals receive the highest doses, not from CT scans or routine diagnostic X-rays but from radioactive interventional procedures [17]. In this case, the doses can be high enough to cause skin and eye crystal damage. The main causes of high doses are the duration of fluoroscopic exposure, the number of films taken, and the use of lower tube voltages in DSA. Radiation interventions can produce both deterministic damage and random radiation effects. Potentially high doses can cause deterministic effects such as erythema or temporary alopecia [18]. Dose issues are therefore not only a general protection issue for professionals and patients but also an integral part of the treatment plan for interventional techniques. Only a well-controlled radiation dose and good radiation protection of patients and professionals can lead to a significant development of interventional techniques. Therefore, as far as interventional technology itself is concerned, radiation dose control and radiation protection are already an important part of interventional technology, and radiation dose is an essential part of the interventional technology treatment planning system.

Theoretical calculations and experimental validation of the in vitro dose levels of these nuclides in the treatment process were carried out to establish a reasonable calculation model and parameters for the estimation of in vitro dose levels. In addition, the cumulative dose distribution in the rooms of patients treated for thyroid cancer during hospitalization was monitored, and finally, specific protection recommendations for patients and exposed personnel were proposed in the light of relevant radiation protection regulations.

## 3. Analytical Design of Nuclear Medicine Exposure Measure Estimation with Computer Intelligent Processing

### 3.1. Intelligent Processing Analysis of Radiometric Computers

In nuclear radiation measurements, processing of the electrical signals generated by and output from the detector is required, including amplification, shaping, screening, analog-to-digital conversion, and analysis of the electrical signals for recording. Front-end electronics are an important part of the detector data readout. However, there are too many summing points, and the longer time to calculate the pulse area may contain too much noise; both will lead to a low signal-to-noise ratio. And the appropriate number of summation points can also reduce the impact of tail accumulation events. According to the characteristics of the detector output signal forming method classification, the preamplifier can be divided into the current-sensitive preamplifier, voltage-sensitive preamplifier, and charge-sensitive preamplifier. The current-sensitive preamplifier is designed as a parallel feedback current amplifier by directly amplifying the current signal from the detector output. The output voltage or current is proportional to the input current [19]. An ideal current-sensitive preamplifier requires a very small input impedance, a very large output impedance, and a good time response and is usually used as a fast amplifier, but the relatively high noise level makes it mainly used in time measurement systems.

Preamplifiers are an important part of signal extraction in both conventional analog and digital energy spectrometry systems. The main challenge in detector electronics is to distinguish small signals from noise. In detector systems, noise is a random signal that is not caused by the physical process to be measured. If the noise only appears at the end of the electronic readout chain, the effect is minimal because the signal is amplified far more than the noise. However, if the noise has appeared in the front part, it may drown out the small signal from the detector output. There are many possible reasons for the appearance of noise, and the noise level can be effectively reduced by careful design of the measurement system, especially the front-end circuitry. The filter not only realizes the low-pass filtering function but also converts the signal from single-ended to differential. To effectively represent the input signal, the amplifier must recover from the load transient and stabilize before the end of the acquisition period. Based on the discussion of preamplifier types, the paper provides design considerations and experimental verification of the front-end circuitry for the strength of the output signal of a *γ*-ray energy measurement detector.

For the weak signal output from the *γ*-ray energy measurement detector, the front-end circuit usually uses a charge-sensitive preamplifier or a current-sensitive preamplifier. The weak signal is highly susceptible to interference from external environmental factors and can even be drowned out, and the sensitivity and measurement accuracy of the measurement circuit of the weak signal will be affected to a large extent. The sensitivity of the circuit depends on the size of the feedback resistance, so to measure smaller signals, we need to increase the feedback resistance, as shown in Figure 1.

The total capacitance of the amplifier input is

(1) $$\begin{array}{c} C_{i}=C_{A}-C_{B}-C_{S}. \end{array}$$

If the input resistance of the amplifier is large, then

(2) $$\begin{array}{c} V_{iM}=\frac{1}{c_{i}}\int_{0}^{tW}i_{D}\left(t\right)\text{d}t. \end{array}$$

This means that the input voltage signal after the input current (*t*) is integrated over the input capacitor is *Vi*, and the signal amplitude *VoM* after passing through the voltage-sensitive preamplifier can be obtained to be proportional to the charge *Q*, and according to the nature of the detector, it yields that the energy of nuclear radiation is proportional to the charge Q. Then, for the voltage-sensitive preamplifier, the charge carried by the current pulse output from the detector is equal, and then, the amplitude of the voltage signal output from this amplifier *V oM* is also equal, independent of the shape of the detector current pulse. It can be seen from the voltage equation that if *Ci* is unstable, it will certainly lead to an unstable amplitude value *VoM* of the output voltage of the voltage-sensitive preamplifier, and the energy resolution of the energy spectrum measurement system will certainly be reduced. As can be seen from the equation of the total capacitance of the amplifier input, instability of its three capacitances is commonly observed, and the stability of the system can be improved if a larger fixed capacitance is connected in parallel at the input.

(3) $$\begin{array}{c} V_{iM}=\frac{1}{c_{i}}\int_{0}^{tW}i_{D}\left(t\right)\text{d}t=\frac{Q}{c_{i}-c_{f}}. \end{array}$$

Preamplifiers are an important part of signal extraction in both conventional analog and digital energy spectrometry systems. The main challenge in detector electronics is to distinguish small signals from noise. In detector systems, noise is a random signal that is not caused by the physical process to be measured. If the noise only appears at the end of the electronic readout chain, the effect is minimal because the signal is amplified far more than the noise. However, if the noise has appeared in the front part, it may drown out the small signal from the detector output. There are many possible reasons for the appearance of noise, and the noise level can be effectively reduced by careful design of the measurement system, especially the front-end circuitry. Based on the discussion of preamplifier types, the paper provides design considerations and experimental verification of the front-end circuitry for the strength of the output signal of a *γ*-ray energy measurement detector.

The short-term stability of the four circuits was tested every 6 hours for a total of 48 hours, and the test data are shown in Figure 2. Compared to the short-term stability test, the gain variation of the circuit under the long-term stability test increased slightly, and the circuit with the protection loop continued to outperform the circuit without the protection loop, where the maximum error of the protection loop single large resistor feedback circuit (LR-R) was -0.464% and the maximum error of the protection loop T-resistor network feedback circuit (TR-R) was -0.178%. The maximum error in the protection loop single large resistor feedback circuit (LR-R) is -0.464%, and the maximum error in the protection loop T-shaped resistor network feedback circuit (TR-R) is -0.178%.

The circuits were tested using a Co source with a radiation intensity of 1.0 Ci, a Cs source at 0.1 Ci, and a Cs source at 20.0 Ci using a gas ionization chamber. An integral nonlinearity of 0.4832% was obtained for a single large resistive feedback circuit with a protection loop and 0.1649% for a T-shaped resistive network feedback circuit with a protection loop. Therefore, the EMI simulation and test prove that the protection loop can shield and protect the circuit, especially for the measurement circuit with high input impedance signal to reduce the adverse effects of input leakage current, EMI, and other interference. The above verification results of the front-end circuit design method provide very meaningful reference data for the design of energy spectrum measurement systems.

In the energy spectrum measurement system, the energy resolution can be used to characterize the system to distinguish the different energies of ions, and it is one of the most important indicators of the energy spectrum measurement system, so we are committed to improving the energy resolution of the system as much as possible. When detecting *γ*-rays, it is desired to have a large detection efficiency for *γ*-rays, to accurately determine the energy of *γ*-rays and to improve the ability to identify *γ*-rays; i.e., the optimal energy spectrum of *γ*-rays needs to be measured. For charged particles with single energy of *E*0, the energy spectrum measured by the energy spectrum measurement system is not a single straight line. For example, a *γ*-ray detector consists of a scintillator detector, a photoelectric converter, and a readout system. If all *γ*-rays deposit all their energy in the scintillator, the readout system will record a pulse height spectrum. We would see peaks at the corresponding locations, a Gaussian curve in the shape of an approximately symmetric bell, and use the full width at half height (FWHM) of the curve as a measure of energy resolution.

(4) $$\begin{array}{c} \eta =\frac{FWHM}{N_{\max}}. \end{array}$$

The smaller the energy resolution *η*, the better; it characterizes the competence of the energy measurement system to separate particles of different energies.

(5) $$\begin{array}{c} \frac{\text{d}q_{st}\left(t\right)}{\text{d}t}=\left(\lambda_{st}-\lambda_{R}\right)q_{st}\left(t\right),\\ \frac{\text{d}q_{si}\left(t\right)}{\text{d}t}=\left(\lambda_{st}-\lambda_{R}\right)q_{st}\left(t\right)+\lambda_{si}q_{st}\left(t\right),\\ \frac{\text{d}q_{ur}\left(t\right)}{\text{d}t}=\left(-\lambda_{st}+\lambda_{R}q_{st}\right)\left(t\right)+\left(1-f\right)\lambda_{si}q_{st}\left(t\right). \end{array}$$

According to the previous discussion, the energy of gamma photons is proportional to the charge of the detector output pulse signal.

(6) $$\begin{array}{c} E\in Q. \end{array}$$

That is, the energy of the gamma photon is proportional to the cumulative sum of discrete data after digitizing the pulse waveform. Therefore, a pulse area calculation algorithm can be used to obtain the energy. However, the noise of the pulse waveform, the overshoot of the falling edge of the pulse, the signal stacking, and the sampling rate of the ADC can affect the accuracy of this algorithm.

In the analog energy spectrum measurement system, the pulse peak is directly extracted through a series of processing of the pulse by analog circuit and then sent to the multichannel pulse amplitude analyzer to extract the relevant digital quantity and then classified statistics, where the spreading effect of the peak hold circuit makes it possible to pick up the maximum value of the pulse at a relatively low sampling rate; in the digital energy spectrum measurement system, there is often only a simple preamplifier before the ADC, or a simple amplification and filtering circuit [20]. On the premise that the patient's urination frequency can be changed, we try to arrange for the patient to take the medicine in the morning of the day and then guide the patient to drink more water and consciously control oneself to increase the frequency of urination to increase the patient's urination frequency on the first day after taking the medicine. In digital energy spectrum measurement systems, there is often only a simple preamplifier before the ADC or a simple amplification and filtering circuit, and after the ADC output, the sampled digital quantities are compared by digital devices such as FPGAs, and the pulse peak is obtained online in real time. And if the ADC sampling rate is high enough, several values near the peak can be selected and averaged to obtain the pulse peak. But there are many high-speed ADCs on the system pressure, but also to consider the subsequent digital signal processing process of calculation speed and storage space requirements, the selected ADC sampling rate cannot be as high as possible.

### 3.2. Nuclear Medicine Exposure Measurement Estimation System Design

The scintillation detector based on silicon photomultiplier Si PM was selected for the detector module, and the system control architecture was determined to be a low-power microcontroller to realize the functions of data processing and system control, etc. Based on the core requirements of high sensitivity, compact structure, and ruggedness, the scintillation detector module was selected. The inherent characteristics of high scintillation crystal density and high atomic number ensure high detection sensitivity; the use of Si PM with higher gain, lower operating voltage, and compact structure replaces the traditional vacuum device photomultiplier, which significantly reduces the size and weight and improves portability with high sensitivity and accuracy; the power supply circuit optimized for Si PM and the choice of low-power microcontroller ensures the overall system. The power supply circuit optimized for the Si PM and the low-power microcontroller ensures the overall low-power consumption of the system and the compact size and easy operation, as shown in Figure 3.

The detector readout circuit converts the current signal from the Si PM output into a voltage signal and connects a spacer circuit to avoid baseline drift that affects the operating state of the subsequent comparison circuit. An ideal current-sensitive preamplifier needs to have a very small input impedance, a large output impedance, and a good time response. The pulse counting circuit uses a comparator to rectify the flicker pulse waveform that exceeds a certain threshold into a logic level pulse that can be easily recognized by the microcontroller and input to the microcontroller for pulse capture [21]. The power supply is a 3.7 V lithium battery, which is supplied to the boost circuit and the regulator circuit to generate the working voltage of the detector, as well as the working voltage and logic high level required for the comparator and the microcontroller to work. Different conversion factors are used for the different energy bands so that the calculated dose contains the effect of energy compensation. When the detector output pulse carries energy information, for example, the amplitude and energy are positively correlated, the energy segmentation can be achieved by amplitude segmentation, which is easier to implement and debug than the above-mentioned scheme of wrapping the compensating material. And because of the large gain of the scintillation detector, the distinction of the signal amplitude corresponding to different energies is greater, which makes it easier to implement the amplitude segmentation method than the silicon semiconductor detector.

The system design requires the use of a material to detect *β*, *X*, and *γ*-rays simultaneously, while *β* detection is more suitable for materials with low effective atomic number *Z* to reduce the detection efficiency due to backscattering of *β*-rays on the surface of the detection material. Therefore, although BGO is more suitable for achieving the detection efficiency and size required in the system design, it is not selected because of its highly effective atomic number, low optical output capability, and poor signal-to-noise ratio due to high refractive index, which affects the detection of low-energy *X*, *β*, and other low-amplitude pulses, as well as its long decay time. The Lu element in LSO is radioactive, which increases the background count of the instrument and affects the minimum detectable dose rate and accuracy of the instrument, so it is excluded from the commonly used cerium-doped silicate crystals. Among YSO and GSO, YSO with a relatively small effective atomic number *Z* is preferred for testing.

In the human respiratory compartment transport model, radionuclides entering the respiratory tract are contoured in two separate ways, partly by particle transport and partly by dissolution and absorption into the blood. In the anterior nasal passage, ET1 compartment, about 1/3 of the deposited material returns to the environment due to the mechanical action of nasal rubbing and breathing, while the remaining 2/3 enters the posterior nasal passage, ET2 compartment, due to swallowing, etc., and then participates in the whole biokinetic process, and due to the lack of blood vessels, it is believed that there is no absorption into the blood in ET1 compartment. A metabolic model with modified parameters applicable to thyroid patients and its computational procedures were used to calculate the activity of the compartments of the stomach, small intestine, blood, thyroid, and the rest of the tissues concerning time. Considering that, for different patients with different thyroidectomies, the thyroid uptake fraction may change, and it was taken to be equal and calculated separately for three cases, as shown in Figure 4.

Looking at equation (6) and its parameter values, it can be found that the formula is divided into two terms, fast and slow exponential terms, in which the share of slow exponential term u2 (0.271) is close to 30% of thyroid uptake fraction in normal subjects, and its corresponding contouring constant (7.41 × 10° min) is also closer to the thyroid contouring rate (6.02 × 109 min'). Therefore, we modified *α* to 0.95 to make the model so modified applicable to patients with thyroid cancer. The front-end circuit usually uses a charge-sensitive preamplifier or a current-sensitive preamplifier. Weak signals are extremely susceptible to interference from external environmental factors or even submerged. The sensitivity and measurement accuracy of weak signal measurement circuits will be greatly affected. To verify the rationality of the above changes, we calculated the time-dependent relationship of urinary 1–131 activity using the MIRD normal model, the MIRD model with modified parameters, and the ICRP I-131 metabolic model (three different thyroid uptake fractions) applicable to patients with thyroid cancer, respectively. As can be seen from the figure, the calculated results of the MIRD normal model were significantly lower than those of the ICRP model applied to thyroid cancer patients, but the MIRD model with modified parameters was very close to the calculated results of the ICRP model with a 5% thyroid uptake fraction. This indicates that the changes to the parameters of the MIRD model in this study are reasonable [22] because the signal is amplified much larger than the noise. However, if noise has already appeared in the front end, it may overwhelm the small-signal output by the detector. Curve fitting, also known as function approximation, is a data processing method that seeks to find the best fit curve for experimental data to obtain more accurate data by analyzing the relevant characteristic parameters of the curve, trying to find the inherent pattern of the data, and using continuous curves to approximate or compare the functional relationship between the coordinates represented by discrete points. Although the curve obtained by “fitting” cannot be guaranteed to pass all sample points, it can be a good approximation of the true value, which can fully reflect the intrinsic relationship between known data and bring great convenience to the analysis of data later.

In the simulation process, it was first found that if the sampling points used for polynomial fitting were taken to points with small signal-to-noise ratios, the fitting effect would be significantly reduced, especially for the baseline sampling points that could not be included. The sampling points used for polynomial fitting are fitted with points with larger signal-to-noise ratios near the peak, so the pulse tail stacking has no effect on the fitting, and this algorithm focuses on the information near the peak of the fitted curve, so the polynomial fitting algorithm is only suitable for peak information extraction and not for waveform recovery. During the simulation experiments of this algorithm, it was found that the start time of the waveform has an important influence on the double exponential function fitting. Comparing the double exponential function fitting of the original waveform and the original waveform fitting with the baseline part removed, the baseline information cannot be included in the fitting process, and if the waveform is fitted from the start point of the pulse waveform, it is almost possible to obtain the original waveform.

## 4. Analysis of Results

### 4.1. Algorithm Performance Results

The trigger rising edge signal and the trigger mask signal are logically spread, and then Cnt_Flag is generated to start the pulse area calculation logic if they are both valid, and the counter Cnt starts counting. To eliminate the nonzero baseline superimposed in the pulse amplitude, the baseline value is estimated using the averaging method, and the baseline of the pulse signal is recovered by deducting the baseline from the pulse amplitude. The average value of the baseline is calculated in the first 4 sampling clock cycles, which is the baseline valuation baseline for this waveform. When solving for the baseline average value, a right shift of 2 bits is used in the FPGA for convenience and efficiency and speed. As can be seen from the ADC sampling waveform graph, the falling edge of the waveform may produce a down-shoot, so after obtaining the baseline, the next data DATA needs to be compared with the baseline. The experiment uses a Na radiation source to irradiate a detector consisting of a single probe LaBr3 single-crystal strip coupled with XP20D0 PMT to finally obtain the energy resolution. The important effect of the choice of the number of accumulated summation points in the algorithm for calculating the pulse area on the energy resolution of the detector at a fixed sampling rate is analyzed, as shown in Figure 5.

From Figure 5, it can be obtained that the energy resolution fluctuates at different pulse start points, and the best energy resolution can be achieved by starting the summation from the 5th point. We test the short-term stability of the four circuits every 6 hours for a total of 48 hours. By testing the number of summation points in the pulse area calculation algorithm, it can be obtained that fewer summation points result in a shorter calculation time and thus fewer photons are collected, while more summation points result in a longer calculation time and may contain too much noise; both result in a low signal-to-noise ratio. And a proper setting of summing points can also reduce the effect of tail stacking events. Therefore, the choice of the number of summing points is crucial for the energy resolution of the detector.

The energy resolution of various energy extraction algorithms was calculated for different sampling rates. The energy resolution of the algorithm for direct pulse peak extraction from the original waveform is 6.62%, and the energy resolution of the algorithm for calculating the pulse area from the original waveform is 5.59%. The energy resolution of each of the other algorithms is shown in Figure 6, and the trend is consistent with the evaluation results of the above simulation.

To solve the problems posed by high-speed ADCs in digital multichannel energy measurement systems, different algorithms are used to achieve the most accurate energy extraction possible at lower sampling rates. The broadening effect of the peak hold circuit enables the maximum value of the pulse to be collected at a relatively low sampling rate; in digital energy spectrum measurement systems, there is often only a simple preamplifier before the ADC. Several algorithms have been simulated and evaluated on the MATLAB platform, and some preliminary conclusions have been obtained. Calculating the energy resolution of each algorithm better corroborates the simulation results and provides a basis for the design and testing experiments of the heavy-ion cancer treatment in-beam PET digital energy spectrometry system.

The inputs can accept single-ended or differential signals. The rail-to-rail differential output and adjustable output common-mode voltage make it ideal for interfacing with differential input ADCs. These ADCs are typically powered from a single supply down to 3 V (2.7 V minimum) and have an optimal common-mode input range close to the intermediate supply. The sampling process of the ADC generates transients caused by the access of the ADC sampling capacitor. The transient temporarily shorts the output of the amplifier as the charge is transferred between the amplifier and the sampling capacitor. For a valid representation of the input signal, the amplifier must recover from this load transient and stabilize before the end of the acquisition cycle. The LTC6605-7 is ready to quickly stabilize from these periodic load pulses. The final filter selects a 6.5 MHz filter with a reference voltage generated by the DAC to map the output signal, which allows a single DC offset to be applied to the common-mode pins. The filter not only implements a low-pass filtering function but also allows the signal to be converted from single-ended to differential, making the signal more resistant to noise during propagation.

### 4.2. Nuclear Medicine Irradiation Measurement Results

The health system has carried out personal dose monitoring since the last century, and the personal dose monitoring rate has been increasing year by year, and the annual effective dose per capita has been decreasing year by year. In particular, the personal dose monitoring rate continues to exceed 90%, and the personal dose monitoring rate has reached 94.5%. There have been 169 personal dose testing institutions reporting data through the system, with data covering 68,342 radiological work-using units and 316,580 monitored people reported by the system. The establishment of the system has played an important role in the improvement of the personal dose monitoring rate and the reduction of annual effective dose per capita. As shown in Figure 7, urine activity in the bladder increases cyclically and then decreases rapidly, with the highest increases in the first two cycles and decreasing amplitude in the subsequent cycles, rapidly decreasing to near 0 within a few days. Cumulative activity in the bladder is mainly contributed by the first day, so it can be expected that the first few cycles are critical in influencing cumulative activity in the bladder and in influencing dose to gonadal organs. In addition to the initial urine volume and bladder urine filling rate, the initial dosing time can be varied in this model.

As the time of dosing approached the time of first urination, the cumulative bladder urine activity, bladder dose, and gonadal organ dose increased significantly. Please rephrase the part for clarity and correctness. the cumulative bladder urine activity increased nearly, both male and female doses increased nearly, the male gonadal dose increased nearly, and the female gonadal dose increased nearly. This may be because if the first urination is too early, the content within the urine at that time is not high, resulting in a poor effect of the first urination. Therefore, patients are advised to urinate after taking the drug to ensure the effectiveness of the first urination. As the time interval between daytime urination on the first day increased, the cumulative bladder urine activity, bladder dose, and gonadal organ dose increased significantly. As the time interval between daytime urination on the first day increased from 1 h to 6 h, the cumulative bladder urine activity increased by nearly 95%, the bladder dose increased by nearly 80% in both men and women, and the gonadal dose increased by nearly 20% in men and nearly 15% in women. However, this effect will not be so significant if the dosing time is delayed, because the shorter the daytime period after dosing, the smaller the number of cycles to increase the frequency and the smaller the effect. Therefore, it is recommended that patients be scheduled to take the drug in the morning of the day as much as possible, provided that the frequency of urination can be changed and then increase the frequency of urination on the first day after taking the drug by directing patients to drink more water and consciously controlling themselves to increase the frequency of urination.

After the data sending and receiving test of each module of the system is completed, the general tuning of the system is carried out. When the host computer and the remote server establish a connection by TCP/IP, the host computer will identify the nuclear radiation detection terminal hardware module and receive the data sent in a certain format, and the host computer will decode it to view the current real-time data. After the host client sets the threshold value for the radiation intensity and temperature of the whole system, and the received nuclear radiation data and temperature are not within this threshold value, the host client program will light up the nuclear radiation intensity alarm indicator or temperature alarm indicator to detect the temperature and radiation intensity of the whole system in the environment in real time and also display the connection status with the remote server in real-time. In the TCP/IP protocol, each time when establishing a long-term connection, the client needs to send packets to the server at regular intervals to notify the server that it is still online, which is a tedious process. When the detector output pulse carries energy information, such as a positive correlation between amplitude and energy, energy segmentation can be realized by amplitude segmentation, which is easier to implement and debug than the above-mentioned solution of wrapping compensation materials. However, if you use HTTP protocol, HTTP is a short connection mechanism established on TCP protocol, which can only upload data. From the perspective of subsequent development, it is necessary to realize the control of the whole onboard nuclear radiation detection terminal by the upper computer client, to better manage the power consumption of the system. Nuclear radiation data and nuclear radiation data graphical display interface are shown in Figure 8.

In this paper, a Microsoft Access database is taken for the storage of the detection data. Database Connectivity Toolset, a toolkit developed by LABVIEW, is used to connect with the data. The column keywords of the table are measurement time, longitude, latitude, height above ground, temperature, radiation intensity, etc. When users query the historical data, they can choose to query the parameters for a certain period. The GPRS communication of the system is tested by using the serial debugging assistant, the transmission of data acquisition of each module of the system is tested by using the network debugging assistant, the real-time display of the data, and the graphical display of the upper computer client program of the whole system is tested, and the historical data storage of the system is tested. The comprehensive test effect of the whole system, the accuracy of data acquisition, and the volume, weight, and power consumption of the system have certain advantages, and it is very easy to be installed on small and medium-sized UAVs, which can achieve the expected effect.

## 5. Conclusion

Based on the contradiction between the need to obtain accurate energy information in the digital measurement system of a heavy-ion cancer treatment device for measuring *γ*-rays in beam PET and the problems caused by the adoption of high-speed ADC in large-scale systems, this thesis investigates the factors influencing energy resolution and the energy extraction algorithm. From the basic composition of the *γ*-ray digital energy measurement system, five main factors are affecting the accurate energy extraction of the *γ*-ray digital energy measurement system. Among them, the selection of ADC of the analog-to-digital converter has a great relationship with it. If many high-speed ADCs are used, there are negative effects on data volume, heat dissipation, system complexity, and cost. It is not practical to use many high sampling rate ADCs in digital energy spectrometry with multiple detector units. The problem of misuse of radiation treatment technology still exists. The awareness of radiation protection among radiation workers in medical institutions is low, especially the health condition of interventional radiology workers is worrying, and the radiation protection of interventional radiology workers needs to be strengthened. We strengthen the personal dose monitoring of internal radiation for nuclear medicine staff; further, we strengthen the supervision and management of radiology treatment institutions, establish a sound system of medical physicists, and improve the radiation health information system.

## Figures and Tables

**Figure 1:** Computerized intelligent processing framework for radiometry.

**Figure 2:** Long-term stability of each circuit.

**Figure 3:** System hardware structure diagram.

**Figure 4:** Variation of activity.

**Figure 5:** Starting point of the scan test 4-channel energy resolution variation graph.

**Figure 6:** Energy resolution of each algorithm.

**Figure 7:** Activity change curve.

**Figure 8:** Graphical display of nuclear radiation data.

## Data Availability

The data used to support the findings of this study are available from the corresponding author upon request.
